# Research on Intelligent Embedded Fan System Based on YOLOv2 Lightweight Algorithm

**DOI:** 10.1155/2022/3484268

**Published:** 2022-07-22

**Authors:** YongHui Wei, KeYu Zhao, XueQiang Lv, JianZhou Feng, HaiJu Hu, Tuyatsetseg Badarch, ZeYu Zhao

**Affiliations:** ^1^LiRen College, Yanshan University, Qinhuangdao, Hebei, China; ^2^School of Information Technology and Design (SITD) Mongolian National University (MNU), Ulan Bator, Mongolia; ^3^Beijing Informat Sci & Technol Univ, Beijing Key Lab Internet Culture Digital Dissemin, Beijing, China; ^4^Yanshan Univ, Sch Informat Sci & Engn,Software Engn Key Lab Hebei Prov, Qinhuangdao, Hebei, China; ^5^School of Economics and Management, Yanshan University, Qinhuangdao, Hebei, China

## Abstract

With the development of artificial intelligence, the application of intelligent algorithms to low-power embedded chips has become a new research topic today. Based on this, this study optimizes the YOLOv2 algorithm by tailoring and successfully deploys it on the K210 chip to train the face object detection algorithm model separately. The intelligent fan with YOLOv2 model deployed in K210 chip can detect the target of the character and obtain the position and size of the character in the machine coordinates. Based on the obtained information of character coordinate position and size, the fan's turning Angle and the size of air supply are intelligently perceived. The experimental results show that the intelligent fan design method proposed here is a new embedded chip intelligent method of cutting and improving the YOLOv2 algorithm. It innovatively designed solo tracking, crowd tracking, and intelligent ranging algorithms, which perform well in human perception of solo tracking and crowd tracking and automatic air volume adjustment, improve the accuracy of air delivery and user comfort, and also provide good theoretical and practical support for the combination of AI and embedded in other fields.

## 1. Introduction

Artificial intelligence is an important part of the future society. It is also a trend of social development to combine home life with artificial intelligence and form a smart home.

Product automation has been developing for more than 70 years since automatic control began after the 1950s as an important means to improve productivity. The concept of smart home emerged in the late 1980s, and people began to have a sense of change from automation to intelligence, but now the so-called smart home, more accurately said should be the Internet of things home, is more inclined to home product interconnection and communication, rather than to give products with intelligence [1, 2]. The current smart home products are not intelligent and have more inclined automation and networking functions. The main reason for this situation is that the traditional embedded chips cannot meet the requirements of high-speed massive numerical computing. Traditional embedded chips are not powerful enough to carry out large-scale parallel computing and run model files generated by deep neural networks. Traditional sensors such as temperature and humidity sensors [3], human infrared sensing sensors, and various gas sensors collect extremely limited information. To gradually transform the traditional automated home or other automation devices into a smart home or smart device, an AI-embedded chip platform that can perform neural network processing is needed [4].

At present, most smart devices work by transmitting photographs, audio, and other data to the cloud server for computing and then returning the computing results to the terminal. Although this way can give full play to the powerful computing power of cloud servers, it makes the devices have a strong dependence on the network, with low real-time performance, and it is not suitable for small intelligent devices with high real-time requirements. How to better combine artificial intelligence technology and hardware products in different fields is a problem worth studying in intelligent product design at this stage [5–8]. The design conducts information collection and feedback through AI, deploys AI model into embedded devices, and upgrades embedded to intelligent embedded, to improve the intelligence of traditional embedded products. Here, we take the design implementation of an intelligent fan product as an example to illustrate the practical significance of this design idea and method.

Today, although air conditioning has entered thousands of households, the traditional electric fans still occupy a large market share. Since the advent of the electric fan, the degree of automation has been continuously improved. The original electric fan canonly supply air in one direction, to the later in a fixed Angle to supply air, and now through the remote control fan switch, speed, and so on [9]. The current electric fan cannot be realized, intelligent judging the distance between people and the fan, automatically adjusting the speed of the fan. And the fan steering cannot change with the change of the person's position. Based on the above analysis of the research situation of home products, intelligent devices, and fans, this study studies this situation in depth, through the YOLOv2-based intelligent embedded fan system lightweight algorithm research, and strives to solve the problem of home intelligent product design [10].

## 2. Related Work

### 2.1. Domestic-Related Work

At present, the fan in the domestic market, for example, household electric fan, has air conditioning fan, intelligent floor fan, leafless fan, etc.

These traditional fan wind speeds on the market cannot be adaptively adjusted when selected, and the air volume cannot be automatically changed when the distance between the user and the fan changes. Part of the fan can shake the head within the set range, but cannot according to the position of the person, and to change the head range of the fan, blowing air does not blow people, resulting in empty waste. Fans in the domestic market generally lack a low degree of intelligence, operation, and adjustment machinery and empty range waste [11].

### 2.2. Foreign-Related Work

As shown in Figure 1, a foreign intelligent fan is composed of fan, power supply circuit, control circuit, infrared remote control sensor, and the swing motor used to make the fan swing, and this intelligent electric fan adopts 8 frequency conversion wind design, low noise, double circulation of the fan blade, 101 cutting airflow, 85° up and down, 60° left and right, the height of three adjustable, the use of the same as natural wind and air supply distance is far, but the fan cannot change with the position of people, follow people to turn.

This fan is a typical representative of the traditional automatic fan, through the cycle execution control program to achieve the set function, and the overall function is still more traditional. Traditional automation can only obtain simple information such as temperature and humidity, but cannot identify and extract relatively complex information such as face and human body [12] and cannot achieve more advanced intelligence of the product based on this information.

## 3. Optimization of the YOLOv2 Model and Correlated Algorithm Design

### 3.1. Based on the Lightweight YOLOv2 Algorithm Process and Working Ideas

YOLOv2 paper full name is as follows: YOLO9000: Better, Faster, Stronger. Although YOLOv1 has a fast detection speed, it is inferior to R-CNN in accuracy, which is not accurate enough in object location and has a low recall rate. YOLO system consists of 24 convolutional layers and 2 fully connected layers. The convolutional layer extracted features, and the fully connected layer predicted the probability of image location and object category. The fully connected layer was removed, so that the SS(B5 + C) structure behind it would stop at the location of 77 channels, and the previous pooling layer was abandoned for the convenience of later calculation. Thus, it can be obtained that this step is the situation of 1313 channels, and it starts to use the RPN of faster R-CNN for reference to select anchor and use anchor to predict the boundary box. So, YOLOv2 has changed the predictable range from 772 to 1313*∗*num_anchors, which has resulted in a huge increase in the number of predictable boxes [13].

The reason why YOLOv2 is selected is that the relatively new model consumes huge memory resources, while YOLOv2, as an early model, consumes less resources, and the work in this study is mainly about object detection and classification [14, 15]. YOLOv2 is enough to meet the requirements and can adapt to the embedded microcontroller with limited resources through clipping [16]. In addition, through experiments, YOLOv3 to YOLOv5 occupy more resources and are difficult to cut, so it is difficult to transplant to the current mainstream embedded chip. Therefore, YOLOv2 model algorithm is selected. The YOLOv2 network can be directly loaded through the KPU module [17] and then combined with the face detection model to realize face recognition [18–20]. The specific programming idea is shown in Figure 2.

The experiment proved that the K210 KPU + YOLO2 + face model can easily realize face detection, and the detection accuracy is very high, and the face detection code is shown as follows [21, 22].

  import KPU as kpu
  import sensor,lcd,time
  from machine import Timer,PWM
  sensor.reset()
  sensor.set_pixformat(sensor.RGB565)
  sensor.set_framesize(sensor.QVGA)
  lcd.Initialize the init () # LCD
  clock = time.clock()
  task = kpu.load(“/sd/facedetect.kmodel”) # Model SD card
  # Model mapping parameters
  anchor = (1.889, 2.5245, 2.9465, 3.94056, 3.99987, 5.3658, 5.155437, 6.92275, 6.718375, 9.01025)
  # Initialize the yolo2 network
  a = kpu.init_yolo2(task, 0.5, 0.3, 5, anchor)
  while(True):
  clock.tick()
  img = sensor.snapshot()
  code = kpu.Run the run_yolo2 (task, img) # on the yolo2 network
  # Show a rectangular representation of a recognized face
  if code:
  for *i* in code:
  print(*i*)
  print(i.rect()[0])
  print(i.x())
  b = img.draw_rectangle(i.rect())
  c = i.rect()[0]

#### 3.1.1. Model Optimization of 3.2 YOLOv2

YOLOv2 is as follows: YOLO 9000: Better, Faster, Stronger [23]. Although YOLOv1 detection speed is fast, YOLOv1 is inferior to R-CNN, which is not accurate in object positioning and has low recall. YOLOv2 abandons dropout, convolves and adds batch normalization, normalizes each layer of the network, improves the convergence speed, performs batch normalization processing, and improves the mAP [18].

YOLOv2 makes the number of predicted boxes more by introducing anchor boxes, and Table 1 is the difference between not introducing anchor boxes and introducing anchor boxes.

Kanzhi K210 is an edge-side AI chip independently developed by Kanan Technology, based on RISC-V architecture and built-in convolutional neural network accelerator KPU.

Model files in H5 format are trained through Keras model library. The h5 file is converted to tflite file, and then, the nncase file is converted to kmodel model. The kmodel model has v3 and v4, and the model is converted with nncase v0.1.0. RC5 is v3 model. v3 has less code, less memory, and high efficiency, but less operators. Finally, the kmodel model was downloaded into the flash of *k* 210 with the following loading code:

  import KPU as kpu
  model_addr_in_flash = 0 × 300000
  task = kpu.load(model_addr_in_flash)
  The model_addr_in_flash here is the offset address of the model in the Flash code = kpu.run_yolo2(task, img)

Images were object-detected by running the YOLOv2 network.

### 3.2. Single-Person Tracking Algorithm Design Based on YOLOv2

Through the YOLOv2 target detection of the image, we can easily get the position coordinates and prediction box size of the target in the image [24]. Through location information, we can obtain the relative position of the target and the camera with the camera as the reference frame. Next, a central position and central area are determined in the image collected by the camera, and the central position is the position of the position coordinates of the target. The central area is the area that determines whether the fan is facing the target. If the position is in this area, it indicates that the fan is facing the target, and if the position is outside this area, the fan needs to control the steering gear, so that the position coordinates of the target coincide with the central area. Coincident means that the fan has been realigned to the target. Therefore, the process of the program is as follows: the face position coordinates obtained by the face detection algorithm are compared with the central position and the central area. When the fan is still and the face position is within the central area, it indicates that the fan is facing the user. When the face position is outside the central area, the deviation between the face position and the central position is calculated, and the rudder is determined according to the deviation size, as shown in Figure 3.

The rotation direction and rotation speed of the machine reduce the deviation to the allowable range. The greater the deviation, the faster the rotation speed, and the smaller the deviation. The fan can quickly track the face and ensure the steering gear, reduce the noise of tracking, and prolong the service life of the steering gear. The flow of steering gear to control the fan is shown in Figure 4.

When running the single-person tracking mode, the fan is initialized and scanned in the rotation range, moving first to the left to the left boundary, then from the left boundary to the right boundary, and then left from the right boundary to the original position. When the fan has not detected the face at the end of an initialization cycle, the initialization cycle procedure is repeated. When the fan detects the face, it jumps to the initialization loop program and runs the single-person tracking algorithm to continuously track the user.

The deviation of the face and camera center and the rotation parameters of the steering gear are as follows.

In the following formula, E is the new gear angle input variable and angle is the current gear angle parameter.

(1) $$\begin{array}{c} E=\left\{\begin{array}{c} angle-0.35,\;\;x<100,\\ angle-0.05,\;100\leq x<120,\\ angle+0.05,\;120<x\leq 140,\\ angle+0.35,\;140<x. \end{array}\right) \end{array}$$

The following code indicates drawing a rectangle when recognizing the face.

  if code:
  for *i* in code:
  print(*i*)
  print(i.rect()[0])
  print(i.x())
  b = img.draw_rectangle(i.rect())
  c = i.rect()[0]
  while(i.rect()[0] < 110 or i.rect()[0] > 130):
  The # *X*-axis reference midline is 120
  The #-------------------------steering gear turns left to the side of-----------------------------
  if (i.rect()[0]) < 100:
  if angle_1 ≥ 2.75:
  angle_1 = angle_1–0.35
  SE_1.duty(angle_1)
  break
  if ((i.rect()[0])≥100 and (i.rect()[0]) < 120):
  if angle_1 ≥ 2.75:
  angle_1 = angle_1–0.05
  SE_1.duty(angle_1)
  Break
  The #-------------------------steering gear turns right for-----------------------------
  if ((i.rect()[0]) > 120 and (i.rect()[0])≤140):
  if angle_1 ≤ 12.45:
  angle_1 = angle_1 + 0.05
  SE_1.duty(angle_1)
  break
  if (i.rect()[0]) > 140:
  if angle_1 ≤ 12.25:
  angle_1 = angle_1 + 0.35
  SE_1.duty(angle_1)
  break
  while(i.rect()[1] < 65 or i.rect()[1] > 85):
  The # *Y*-axis reference center line 75
  # The smaller the duty cycle, the rudder engine back; portrait up, the smaller the *y* value
  #------------------------------steering up-----------------------------
  if (i.rect()[1]) < 45:
  if angle_2 ≥ 2.75:
  angle_2 = angle_2–0.25
  SE_2.duty(angle_2)
  break
  if (i.rect()[1])≥45 and (i.rect()[1]) < 75:
  if angle_2 ≥ 2.75:
  angle_2 = angle_2–0.05
  SE_2.duty(angle_2)
  Break
  #------------------------------steering under-----------------------------
  if (i.rect()[1]) > 105:
  if angle_2 ≤ 11.65:
  angle_2 = angle_2 + 0.25
  SE_2.duty(angle_2)
  break
  if (i.rect()[1])≤105 and (i.rect()[1]) > 75:
  if angle_2 ≤ 12.45:
  angle_2 = angle_2 + 0.05
  SE_2.duty(angle_2)
  break

### 3.3. Design of the Crowd Tracking Algorithm

When the fan faces multiple users, it can achieve accurate air supply within the crowd range through the crowd tracking algorithm. The specific idea of the algorithm is as follows.

First, the fan controls the horizontal steering gear from left to right, and when the fan first identifies the user and the user is in the middle of the fan, the current fan orientation of the angle is recorded, which is the left boundary of the crowd. Then, the fan continues to rotate from left to right. When the fan recognizes the user again and the user is in the middle of the fan field, the orientation angle of the current fan is the right boundary. This step is repeated to update the right boundary position in real time until the initialization scan is completed. The flow chart of crowd tracking algorithm is shown in Figure 5.

When the left boundary of the fan reaches the left boundary, the camera detects whether the fan is to the left of the fan, records the current steering angle as the new left boundary, and then controls the steering machine to turn right. When turning right to the right boundary, the above procedure is performed.

### 3.4. Design of Wind Volume Dynamic Adjustment Algorithm

#### 3.4.1. Calculation of Human-Fan Distance

The dynamic air volume adjustment of fans first calculates the distance between human fans through visual ranging and then controls the speed of the fan motor based on different distances, to realize the dynamic adjustment of the air volume with the distance between people and fans, so that the body sensing air volume blowing to the user remains relatively constant.

As one of the basic technologies in the field of machine vision, visual ranging has been widely paid attention to. It plays an important position in the field of robot and is widely used in machine vision positioning, target tracking, visual obstacle avoidance, etc. Machine vision measurement is mainly divided into monocular visual measurement, binocular visual measurement, and multilocular visual measurement. The synergy between cameras in binocular and multilocular systems is not well controlled, and the monocular visual system can overcome the aforementioned synergy between cameras. In terms of production cost, monocular vision is more cost-saving than binocular and binocular systems. Monocular visual ranging has the advantages of simple structure, fast computing speed, and low cost, which is suitable for scenes with low-ranging accuracy requirements. Therefore, this design adopts single-visual distance to human distance measurement.

The principle of single-visual ranging is similar to that of pore imaging.

As shown in Figure 6, assume a target or object of width W. This target is placed at a *D* distance from the camera. The object is photographed with a camera and the pixel width P of the object is measured.

This gives the following formula for the focal length of the camera:

(2) $$\begin{array}{c} F=\frac{\left(P\times D\right)}{W}. \end{array}$$

When continuing to move the camera near or away from the object or target, you can use a similar triangle to calculate the distance of the object from the camera:

(3) $$\begin{array}{c} D\prime =\frac{\left(W\times F\right)}{P}. \end{array}$$

Thus, if the focal length of the camera and the size of the target object are known, the distance between the targets to the camera can be obtained according to the formula (2). The fan wind speed can be adjusted according to the distance.

By measuring the size of several groups of prediction frames and the data of the distance between the human fan and the prediction frame, the function of the distance between the human fan and the prediction frame is constructed to calculate the distance between the human fan and the prediction frame. As shown in Table 2, the prediction box and fan distance function are built to realize the fan distance estimation, and the figure is the prediction box pixel width (W), pixel height (H), pixel diagonal length (*X*), and fan distance (Y).

By curve fitting the data in Table 2 with MATLAB, Figure 7 and Formula 4 can be obtained as follows:

(4) $$\begin{array}{c} f\left(x\right)=p1\times x^{3}+p2\times x^{2}+p3\times x+p4. \end{array}$$

In particular, *p*1 = −4.055e-05, *p*2 = 0.01971, *p*3 = −3.203, and *p*4 = 196.6; according to formula (4), we can draw from the diagonal of the prediction box the distance between the target and the camera. The calculation of human-fan distance is realized.

According to the X-Y function curve in the above figure, the human-fan distance Y can be estimated through the diagonal *X* of the prediction box, to adjust the air volume.

#### 3.4.2. Dynamic Adjustment Algorithm of Wind Volume

The essence of air volume control is to control the motor speed. According to the different working power supplies, the motor can be divided into DC motor and AC motor. There are two common methods to change the rotation speed of the AC motor: the first is to change the frequency of the alternating current at the input end, which can be achieved through the frequency converter; the second is to change the rotation speed at the output end, that is, to change the gear speed of the AC motor in proportion, which can be achieved through the deceleration box. For a DC motor, its power supply voltage is a DC input, which can be controlled by PWM technology.

Considering the simple speed regulation mode of the DC motor, the wide range of adjustable speed, more air shift, soft wind, farther air supply distance, and the use of the DC motor, with better silent fan effect and energy-saving effect, this design adopts the DC motor.

In terms of motor drive, the motor drive module is selected as TB6612FNG for this design. The dual-way DC motor drive is based on TB6612FNG drive IC design and adopts a special logical control mode, and only 4 tube feet can realize dual-way motor control, saving valuable IO resources.

PWM is the abbreviation of pulse width modulation. It is the number of analog signal levels by modulating the width of a series of pulses, equivalent to the required waveform. Pulse width modulation is a very effective technique that uses the digital output of microprocessors to control analog circuits, which is widely used in many fields, from measurement and communication to power control and transformation.

Changes in the duty cycle of the PWM can regulate changes in signal, energy, etc. The duty cycle refers to the percentage of the signal at high level in the whole signal cycle. For example, the duty cycle is 50%.

PWM speed regulation is to adjust the duty ratio to simulate different voltage values, so as to control the voltage at both ends of the motor to achieve speed regulation.

The K210 contains 3 timers with 4 channels available for each timer. This design enables the motor speed regulation through the following functions:

  def PWM_WindSpeed(*i*):
  tim = Timer(Timer.TIMER0, Timer.CHANNEL0, mode = Timer.MODE_PWM)
  pwm = PWM(tim, freq = 10000, duty = 100, pin = 12)
  pwm.duty(*i*)
  SE_3.duty(fan_speed)

The fan_speed here represents the duty cycle parameter.

To make the wind volume change dynamically according to the change in the fan distance, the closer the fan distance, the smaller the fan distance, the larger the fan, and the distance between the fan and the difference, and considering the different requirements for fan gear, the gear should also be one of the input quantities of the air volume dynamic regulation algorithm. First, all possible values for the predicted human-fan distance were normalized, with the normalized values multiplied by the 60% motor duty cycle. At this point, the duty cycle obtained between 0% and 60% is the duty cycle that can be dynamically adjusted according to the human-fan distance. To combine the gear and the air volume, the remaining 40% duty cycle is divided into two gears, and 20% is superimposed on the original duty cycle to realize the fan motor speed based on the dynamic adjustment of the fan distance. To facilitate debugging, a bias item PT_x is superimposed on each output. If the air volume at this position is slightly different from that expected, it can be adjusted through the bias item:

(5) $$\begin{array}{c} \mathrm{Output}=\frac{y}{y\_\max}\times 60+\left(tap\_position-1\right)\times 20+PT\_x. \end{array}$$

Here, *y* is the diagonal length of the input prediction box, *y* _max is the maximum value that the diagonal can take, and tap_position is the selected block. Since a target has nine possible prediction boxes, there are nine different biases; namely, each prediction box corresponds to one PT_x.

#### 3.4.3. Hardware Design of Intelligent Fan

The hardware part of the fan consists of K210 core board, motor drive module, Bluetooth module, and steering machine [25–28]. In addition to the work of the traditional embedded SCM, K210 is also responsible for the object detection of objects. The K210 controls the motor of the fan through the motor drive module and controls the speed of the fan by exporting different PWM waves. The Bluetooth module realizes the communication between the fan and the mobile phone [29, 30], so that users can easily control the fan and switch the mode through the mobile phone, and the module circuit diagram is shown in Figure 8.

As shown in Figure 9, the face detected the wind based on K210.

The fan has a good recognition effect and can track the movement of the user stably. After testing, the image recognition speed on the K210 device is 11 frames/s, enough to ensure the normal operation of the system.

## 4. Conclusions and Future Work

This study presents a lightweight algorithm study of intelligent embedded fan system based on YOLOv2 and discusses and analyzes the current situation, existing problems, and solutions of traditional smart home products. In this paper, YOLOv2 target detection algorithm is deployed on Kanzhi K210 chip. Combined with single person tracking algorithm, crowd tracking algorithm, and dynamic air volume adjustment algorithm, the intelligent fan realizes the real-time tracking of individual position changes, as well as the real-time tracking of crowd range, and accurate air supply. The air volume can be dynamically adjusted according to the distance between the user and the fan. The experimental results show that the algorithm can improve the accuracy of fan and realize the intelligence. However, there are some remaining problems in the content of this study, which need further analysis. In the current recognition process, limited by the size of the model input image, only 224224 images are identified, reducing the success rate of target detection in a complex environment. The K210 has 6 MB universal RAM and 2 MB KPU dedicated RAM, which can only load about 4 MB of models when running MaixPy code, requiring pruning optimization for too large models. Follow-up work will continue to optimize the target detection and pruning algorithms. At the same time, in the subsequent research, we will focus on the application of other AI algorithms in embedded systems, to improve the efficiency and accuracy of execution, and further expand the new ideas of lightweight AI algorithms.

This study provides a good example of the lightweight transplantation of AI algorithms into embedded systems. With the development of artificial intelligence chips, it will become easier and easier to deploy neural networks to embedded chips. Now, the mainstream AI development boards are Jetson Nano, Jetson TX2, K210, etc. These AI development boards enable object recognition, object detection and tracking, speech recognition, and other visual development functions. Based on these features, and with the full imagination, we can develop more interesting and more powerful smart products.

## Figures and Tables

**Figure 1:** American shule air circulation fan.

**Figure 2:** Flow chart of the model deployment.

**Figure 3:** Fan obtains different locations relative to the visual center.

**Figure 4:** Flowchart of steering gear control fan.

**Figure 5:** Flow chart of the population tracking algorithm.

**Figure 6:** Schematic diagram of single-visual ranging.

**Figure 7:** Plot of a function of prediction box size and fan distance.

**Figure 8:** Module circuit diagram.

**Figure 9:** Model.

**Table 1:** With or without anchor comparison.

Without anchor	69.5 mAP	81% recall
With anchor	69.2 mAP	88% recall

**Table 2:** Data table of target detection and prediction box size and human-fan distance.

W	H	X	Y
135	181	226	12
107	144	179	20
82	111	138	25
64	86	107	30
47	79	92	40
38	63	74	50
37	50	62	60
30	40	50	80
24	32	40	90

## Data Availability

The data used to support the findings of this study are available from the corresponding author upon request.
